The article "The long non-coding RNA ASMTL-AS1 promotes hepatocellular carcinoma progression by sponging miR-1343-3p that suppresses LAMC1 (laminin subunit gamma 1)" was retracted in 2023. Reasons: original data or images not available; unreliable results or conclusions; concerns about the data; concerns about the results or conclusions.

# The long non-coding RNA ASMTL-AS1 promotes hepatocellular carcinoma progression by sponging miR-1343-3p that suppresses LAMC1 (laminin subunit gamma 1)

**DOI:** 10.1080/21655979.2021.2012628

**Published:** 2021-12-29

**Authors:** Yanjie Mou, Qinguo Sun

**Affiliations:** Traditional Chinese Medicine, Wuhan Third Hospital (Tongren Hospital of Wuhan University), Wuhan, Hubei, China

**Keywords:** Cerna, proliferation, migration, lncRNA

## Abstract

Long non-coding RNAs (lncRNAs) are critical regulators of hepatocellular carcinoma (HCC) carcinogenesis and development. We aimed to identify the function of the lncRNA ASMTL-AS1 during HCC malignancy. The expression of ASMTL-AS1, miR-1343-3p, and LAMC1 (laminin subunit gamma 1) was assessed in HCC tissues and cells. Cell Counting Kit-8 (CCK8) and Transwell migration assays were performed to determine the effect of ASMTL-AS1 on HCC cell proliferation and migration. Cell apoptosis was identified by detecting Bax and Bcl-2 protein expression using Western blotting, and a xenograft assay was performed to investigate tumor growth *in vivo*. The interplay between miR-1343-3p and ASMTL-AS1 or LAMC1 was verified through luciferase reporter and RNA immunoprecipitation assays. ASMTL-AS1 and LAMC1 were highly expressed in HCC tissues and cells, whereas miR-1343-3p showed low expression. Clinically, miR-1343-3p expression in HCC tissues showed a negative correlation with ASMTL-AS1 or LAMC1 expression. Functional assays demonstrated that ASMTL-AS1 silencing suppressed HCC cell proliferation and migration and increased cell apoptosis. More interestingly, ASMTL-AS1 sponged miR-1343-3p and miR-1343-3p to target the 3ʹ-UTR of LAMC1, thereby interfering with the malignant behavior of HCC cells. In conclusion, ASMTL-AS1 acts as a carcinogen in HCC through competing endogenous RNA (ceRNA) activity in the miR-1343-3p/LAMC1 axis. Our findings demonstrate that regulating ASMTL-AS1/miR-1343-3p/LAMC1-mediated HCC cell malignancy might be an effective method to interfere with HCC progression.

## Introduction

Hepatocellular carcinoma (HCC) is a highly malignant type of digestive system cancer [1]. According to global cancer statistics, in 2020, 905,677 new HCC cases were diagnosed, and 830,180 HCC-related deaths occurred. Tremendous progress in surgery and radiochemotherapy has improved the clinical outcomes of patients with early-stage disease [2]. However, HCC is frequently diagnosed later, and current treatment modalities have limited efficacy [3]. Therefore, understanding the underlying mechanism by which HCC progresses is critical for exploring effective diagnostic and therapeutic targets for HCC.

Long non-coding RNAs (lncRNAs) are a group of RNA transcripts that are longer than 200 nucleotides. Due to their lack of protein-coding potential, they were initially defined as transcriptional noises without biological functions. Nevertheless, their abundance in the mammalian genome and various coding-independent functions enable them to be actively implicated in different cellular processes [4,5]. Apart from the aberrant expression of protein-coding genes, dysregulation of lncRNAs, like other non-coding RNAs, is critical in tumorigenesis and cancer progression [6]. For example, lncRNA-PDPK2P is upregulated in HCC tissues and negatively associated with the clinicopathological features of HCC patients [7]. The lncRNA CSMD1-1 hyperactivates oncogenic phosphatase and tensin homolog deleted on chromosome ten signaling, thereby enhancing the malignant phenotypes of HCC cells [8]. The lncRNA CSMD1-1 enables HCC malignancy by blocking the ubiquitin-proteasome degradation pathway of MYC and increasing MYC expression, which favors HCC progression [9].

Among the multiple mechanisms by which lncRNAs interfere with gene expression, the competing endogenous RNA (ceRNA) mechanism has always been a research hotspot. ASMTL-AS1 has been reported to act as a tumor suppressor in thyroid carcinoma [10] and breast cancer [11] due to its ceRNA activity. However, a recent study showed that ASMTL-AS1 is highly expressed in HCC and favors malignant tumor phenotypes through miR-342-3p/YAP (Yes1-associated transcriptional regulator) signaling [12]. It is widely accepted that lncRNAs can bind different miRNAs and construct complex regulatory networks [13]. Therefore, we aimed to further validate the role of ASMTL-AS1 in HCC *in vitro* and *in vivo*.

Using bioinformatics analysis, we hypothesized that the ASMTL-AS1/miR-1343-3p/laminin subunit gamma 1 (LAMC1) axis plays a role in HCC progression. We conducted a series of functional assays to validate the ceRNA mechanism during HCC malignancy to support this assumption. Hence, our findings may enrich our understanding of ASMTL-AS1 involvement in HCC progression.

## Methods

### Bioinformatics analysis

Gene Expression Profiling Interactive Analysis (GEPIA, http://gepia.cancer-pku.cn/index.html) stored the mRNA expression data of HCC samples and normal samples. With an adjusted P < 0.05 and logFC ≥ 2, the upregulated differentially expressed genes (DEGs) in HCC samples were screened out. At the same time, starBase (https://starbase.sysu.edu.cn/index.php) was used to predict the target mRNAs of miR-1343-3p. Finally, the common mRNAs in GEPIA and starBase were overlapped using Venny 2.1.0 (https://bioinfogp.cnb.csic.es/tools/venny/).

### Tissue samples

From January 2018 to January 2020, 36 HCC tissues and paired paracancerous tissues from fresh surgical specimens were obtained from patients with HCC who had received surgical therapy at the Wuhan Third Hospital. All patients signed a written consent form to participate in this study. The tissues were used following ethics approval granted by the Institutional Ethics Committee of Wuhan Third Hospital (LW2019-070). All clinical samples were kept at −80°C for gene quantification.

### Cell culture

Normal human liver epithelial cells (THLE2), HCCLM3, Hep3B, Huh7, and SNU-182 liver cancer cells were purchased from the Cell Bank of the Chinese Academy of Sciences (Shanghai, China). THLE2, HCCLM3, and Huh7 cells were grown in DMEM medium, Hep3B in MEM medium, and SNU-182 in RPMI-1640 medium. All cells were maintained at 37°C in a humidified incubator with 5% CO_2_.

### Cell transfection

For ASMTL-AS1 knockdown, pre-designed siRNAs targeting ASMTL-AS1 (si-ASMTL-AS1) or LAMC1 (si-LAMC1) and their corresponding negative control (si-NC) were provided by Genepharma (Shanghai, China). The miR-1343-3p mimic, miR-1343-3p inhibitor, mimic-NC and inhibitor-NC were also provided by Genepharma. All cell transfections were performed using Lipofectamine 3000 reagent (Life Technologies, USA). Forty-eight hours post-transfection, HCCLM3 and Huh7 cells were subjected to the following assays.

### Real-Time quantitative reverse transcription PCR (qRT-PCR)

To examine ASMTL-AS1, miR-1343-3p, and LAMC1 expression in HCC tissues or cells, TRIzol reagent (Thermo Fisher, USA) was used to isolate total RNA. The RNA was subjected to reverse transcription reactions to construct cDNA using a high-capacity cDNA reverse transcription kit (Applied Biosystems, USA). A OneStep RT–PCR kit (Qiagen, China) was used for qRT-PCR. Relative transcript abundance was obtained using the 2−∆∆CT method [14], normalizing to U6 and β-actin expression. The primers used for qRT-PCR are listed in Table 1.

**Table 1.** The sequences of the primers in this study

Primer	Sequences
ASMTL-AS1	Forward: 5′-TGACAGTCTCTGCACCAAGG-3′
	Reverse: 5′-CTCAGTCCTTCTCCGCACTC-3′
LAMC1	Forward: 5′-CACTGGCTGGTTACACTTTACCTCT-3′
	Reverse: 5′-CCTTTTGAGTCCTAATGTCCAAGAC-3′
miR-1343-3p	Forward: 5ʹ-CTAGTGCAGTTGTGACTCTACCCAGGAAA-3’
	Reverse: 5ʹ-AGCTTTTCCTGGGTAGAGTCAACTGCA-3’
GAPDH	Forward: 5ʹ-GGAGCGAGATCCCTCCAAAAT-3’
	Reverse: 5ʹ-GGCTGTTGTCATACTTCTCATGG-3’
U6	Forward: 5ʹ-TGCGGGTGCTCGCTTCGGC-3’
	Reverse: 5ʹ-CCAGTGCAGGGTCCGAGGT-3’
NAME	FROM
**ASMTL-AS1**	Forward: 5′-TGACAGTCTCTGCACCAAGG-3′
	Reverse: 5′-CTCAGTCCTTCTCCGCACTC-3′
**LAMC1**	Forward: 5′-CACTGGCTGGTTACACTTTACCTCT-3′
	Reverse: 5′-CCTTTTGAGTCCTAATGTCCAAGAC-3′
**miR-1343-3p**	Forward: 5’-CTAGTGCAGTTGTGACTCTACCCAGGAAA-3’
	Reverse: 5’-AGCTTTTCCTGGGTAGAGTCAACTGCA-3’
**GAPDH**	Forward: 5’-GGAGCGAGATCCCTCCAAAAT-3’
	Reverse: 5’-GGCTGTTGTCATACTTCTCATGG-3’
**U6**	Forward: 5’-TGCGGGTGCTCGCTTCGGC-3’
	Reverse: 5’-CCAGTGCAGGGTCCGAGGT-3’

### Western blot analysis

Cell lysates were obtained using radioimmunoprecipitation assay buffer (Beyotime, China). After microcentrifugation, the supernatant was subjected to dose assessment using a BCA protein quantitative kit (Hualikexi, China). Equal amounts of protein were loaded onto a 10% SDS-PAGE following electrophoresis. Following membrane transfer, the membrane was blocked with 5% nonfat milk for 30 min at room temperature. Anti-Bax (1:1000, cat: 33–6400, Thermo Fisher), anti-bcl-2 (1:1000, cat: MA5-11757, Thermo Fisher), anti-LAMC1 (1:1000, cat:PA5-36300, Thermo Fisher), and anti-GAPDH (1:1000, cat:MA1-16757, Thermo Fisher) antibodies were used to label the proteins on the membranes in a cool room overnight. Subsequently, secondary antibodies were used to detect the target proteins on the membranes. The Pierce ECL Western blot substrate was used for staining.

### Cell Counting Kit-8 (CCK8) assay

HCCLM3 and Huh7 cells (5000 cells/well) were plated in 96-well plates. After incubation for 24, 48, 72, and 96 h, the cells were treated with 10 μL CCK8 reagent for 30 minutes. The absorbance at 450 nm was then read using an ELISA plate reader (Biotek, USA) as described before [15].

### Transwell migration assays

Cells (1 × 10^5^) were placed in the upper compartment of Millicell cell culture inserts (Merck KGaA, Germany) positioned on a 24-well companion plate. After incubation for 36 h, the inserts were fixed with 4% paraformaldehyde for 15 min and then stained with crystal violet for an additional 15 min. After removing the non-invading cells, the invading cells were counted under a microscope and captured as reported previously [16].

### Subcellular fractionation

A nucleus-cytoplasm separation PARIS Kit (Thermo Fisher Scientific, USA) was employed following the manufacturer’s instructions to isolate nuclear fractions from the cytoplasmic fractions of HCC cells. Next, total RNA was isolated and purified for qRT-PCR analysis.

### Luciferase assay

The fragments of LAMC1 3ʹ-UTR and ASMTL-AS1 carrying the putative binding site of miR-1343-3p and the corresponding mutant sequence were inserted into a pmirGLO luciferase vector to establish luciferase reporter vectors: ASMTL-AS1-WT, LAMC1 3ʹUTR WT, ASMTL-AS1-MUT, and LAMC1 3ʹUTR MUT. These constructed luciferase vectors were introduced into HCCLM3 and Huh7 cells at approximately 75% confluence, accompanied by a miR-1343-3p mimic or NC. Forty-eight hours post-transfection, luciferase signals were examined using a dual-luciferase reporter assay system. Luciferase activity was calculated as firefly luciferase activity/Renilla luciferase activity [17].

### Ago2-RNA immunoprecipitation

To verify the interaction between ASMTL-AS1 and miR-1343-3p, Ago2-RNA immunoprecipitation was conducted in HCCLM3 and Huh7 cells with miR-1343-3p mimic or NC using a Nuclear RNA-Binding Protein Immunoprecipitation Kit (Sigma-Aldrich, USA), as described previously [18]. Briefly, transfected HCC cells were exposed to a harsh lysis buffer for 30 min. After microcentrifugation, the supernatant was collected and incubated with pre-prepared protein A magnetic beads with anti-Rat IgG or Anti-Rat-AGO2. After 30 min of incubation, immunoprecipitated complexes on a magnetic stand were collected and diluted for RNA quantification.

### Xenograft assay

All animal experiments were approved by the Institutional Animal Care and Use Committee of the Wuhan Third Hospital. Hepatocellular carcinoma xenograft tumors were triggered in 10 BALB/c nude mice (male, 5-week old) purchased from the Wuhan University Center for Animal Experiments/Animal Biosafety Level III laboratory (ABSL-III lab) of Wuhan University (Wuhan, Hubei, China). Each mouse was kept individually with free access to food and water. Huh7 cells transfected with Sh-ASMTL-AS1 or Sh-ASMTL-AS1-NC (Gema, China) were subcutaneously administered to the mice to initiate xenograft tumors. After subcutaneous implantation, a Vernier caliper was used to measure the size of the xenograft tumors every 4 days. The mice were euthanized via CO_2_ inhalation at 28 days post-injection and the tumor weights were recorded.

### Statistical analysis

GraphPad 9.0 software was applied for data analysis. All results were presented as the mean ± standard deviation. Paired Student’s t-test was applied to analyze the variables from two groups, while analysis of variance (ANOVA) was used to analyze the variables from multiple groups. Spearman’s analysis was adopted to evaluate the correlation between miR-1343-3p, ASMTL-AS1, and LAMC1. Statistical differences were determined when P < 0.05.

## Results

We aimed to further validate the role of ASMTL-AS1 in HCC *in vitro* and *in vivo*. Using bioinformatics analysis and a series of functional cell assays, we identified an ASMTL-AS1/miR-1343-3p/LAMC1 ceRNA network that regulates HCC progression.

### Role of the ASMTL-AS1/miR-1343-3p/LAMC1 axis in HCC

Since the ceRNA activity of ASMTL-AS1 has been reported in HCC, we intended to find another downstream axis of ASMTL-AS1 in HCC. According to the starBase database, ASMTL-AS1 has three target miRNAs: miR-1343-3p, miR-6783-3p, and miR-342-3p. Among them, we found that miR-1343-3p had not been studied in HCC; thus, we chose this miRNA for further experiments. By intersecting the target mRNAs of miR-1343-3p using starBase and the DEGs from GEPIA data, six genes were identified: *CD34, LAMC1, TROAP, MCM2, AURKB*, and *CD74* (Figure 1). Among them, *LAMC1* was of interest because of its oncogenic role in HCC. However, whether ASMTL-AS1 and miR-1343-3p can regulate LAMC1 in HCC remains to be further studied.

**Figure 1.** ASMTL-AS1/miR-1343-3p/LAMC1 axis was selected to be studied in HCC. a. A Venny diagram showing the overlapping genes of the target mRNAs of miR-1343-3p by starbase database and the DEGs from GEPIA LIHC (liver hepatocellular carcinoma) data. DEG: differentially expressed genes. Selection criteria: adjusted P < 0.05, logFC≥2.

### ASMTL-AS1 silencing retards HCC progression

ASMTL-AS1 transcript levels in HCC cells were higher than those in THLE2 cells (Figure 2(a)). In particular, an almost 2-fold increase in ASMTL-AS1 transcript levels was detected in HCCLM3 and Huh7 cells. Hence, both HCC cells were selected for subsequent *in vitro* assays. Similarly, ASMTL-AS1 transcript levels also showed the same elevation in HCC tissues compared to paired normal tissues (Figure 2(b)). Furthermore, preferential cytoplasmic localization of ASMTL-AS1 was observed in HCCLM3 and Huh7 cells (Figure 2(c)), suggesting a regulatory role for ASMTL-AS1 in HCC. To further determine its biological function, we first introduced si-ASMTL-AS1 and si-NC into HCCLM3 and Huh7 cells to establish ASMTL-AS1-silence HCC cells (Figure 2(d)), as evidenced via qRT-PCR analysis. Subsequent CCK8 assays demonstrated a lower proliferative rate of ASMTL-AS1-silence HCC cells than that of the control HCC cells (Figure 2(e)). These results were substantiated through Western blot analysis, which demonstrated that ASMTL-AS1 silencing increased the expression of the pro-apoptotic protein Bax and decreased the expression of the anti-apoptotic protein Bcl-2 (Figure 2(f)). The results of the Transwell migration assays illustrated that ASMTL-AS1 downregulation resulted in the impairment of HCC cell migration (Figure 2(g)). The xenograft assay revealed that silencing ASMTL-AS1 inhibited tumor growth *in vivo* (Figure 2(h)). All findings suggested that ASMTL-AS1 functioned as a tumor promoter to increase the proliferation and migration of HCC cells *in vitro* and retarded tumor growth *in vivo*.

**Figure 2.** ASMTL-AS1 downregulation inhibits HCC proliferation and migration in vitro. a. qRT-PCR analysis of ASMTL-AS1 expression in HCC cell lines and THLE2 cells. b. qRT-PCR analysis of ASMTL-AS1 expression in HCC tissues and normal tissues. c. ASMTL-AS1 mainly located in cytoplasm. d. The effects of transfection of siASMTL-AS1 and si-NC in HCC cell lines (HCCLM3 and Huh7 cells) were detected by PCR analysis. e. CCK-8 assay was performed to test the cell viability and proliferation in downregulated CASMTL-AS1 groups (si-ASMTL-AS1) and negative control group (si-NC). f. Western blotting analysis was performed to detect the Bax and Bcl-2 expression in HCCLM3 and Huh7 cells. G. Transwell assay was performed the migrated and invaded abilities in HCC cell lines. * P < 0.05, ** P < 0.001, vs. Si-NC. H. ASMTL-AS1 downregulation inhibited HCC tumor growth in vivo. ** P < 0.001, vs. Sh-NC.

### ASMTL-AS1 binds to miR-1343-3p to modulate its expression

Since there is predominant cytoplasmic localization of ASMTL-AS1 in HCC cells, we further investigated the ceRNA network in HCC cells. As indicated by the starBase prediction, ASMTL-AS1 shared a complementary sequence with miR-1343-3p (Figure 3(a)). Furthermore, transfection with the miR-1343-3p mimic resulted in reduced ASMTL-AS1 WT-mediated luciferase activity, while the mutant ASMTL-AS1 sequence had abrogated luciferase activity (Figure 3(b)). Following anti-AGO2 RNA immunoprecipitation (RIP) assays, a noticeable enrichment of ASMTL-AS1 in the AGO2-immunoprecipitated complex was detected in HCC cells transfected with the miR-1343-3p mimic (Figure 3(c)). Accordingly, we further evaluated miR-1343-3p expression in HCC tissues. Undoubtedly, a decrease in miR-1343-3p expression was detected (Figure 3(d)). Interestingly, miR-1343-3p expression was negatively correlated with ASMTL-AS1 expression in HCC tissues (Figure 3(e)). In HCCLM3 and Huh7 cells, we found the same low expression of miR-1343-3p (Figure 3(f)). To further explore whether ASMTL-AS1 is responsible for miR-1343-3p downregulation in HCC cells, we transfected HCC cells with si-ASMTL-AS1, miR-1343-3p inhibitor, or their NCs. The subsequent qRT-PCR analysis demonstrated that si-ASMTL-AS1 transfection increased miR-1343-3p expression, which was abrogated by additional transfection of miR-1343-3p inhibitor (Figure 3(g)). These data suggest that ASMTL-AS1 sponges miR-1343-3p and downregulates miR-1343-3p expression.

**Figure 3.** ASMTL-AS1 binds to miR-1343-3p to modulate its expression. a. Schematic diagram of the complementary sequence between ASMTL-AS1 and miR-1343-3p. b. Luciferase reporter assay revealed the relationship between miR-1343-3p and ASMTL-AS1. c. An anti-AGO2 RIP assay was performed in HCCLM3 and Huh cells after transfection with miR-1343-3p mimics or mimic NC, followed by qRT-PCR. d. qRT-PCR analyzing the miR-1343-3p in HCC tissues. e. Pearson’ correlation between miR-1343-3p and ASMTL-AS1. f. qRT-PCR analyzing the miR-1343-3p in HCC cells. g. The relative miR-1343-3p and ASMTL-AS1 expression was detected after HCCLM3 and Huh cells transfected with si-NC, si-ASMTL-AS1, miR-1343-3p inhibitor, inhibitor NC, si-ASMTL-AS1+ miR-1343-3p inhibitor. * P < 0.05, ** P < 0.001, vs.Si-NC; #P < 0.05, ## P < 0.001, vs.inhibitor-NC; ΔP<0.05, ΔΔP<0.001, vs. si-lnc+inhibitor.

### MiR-1343-3p inhibitor abrogates the deceleration of HCC cell proliferation and migration caused by ASMTL-AS1 silencing

Cell functional assays were performed to verify whether ASMTL-AS1 oncogenicity is dependent on miR-1343-3p downregulation. As shown in Figure 4(a), anti-miR-1343-3p treatment augmented HCC cell proliferation, yet the promoting effect was almost eliminated upon ASMTL-AS1 silencing. Likewise, the anti-apoptotic effect of the miR-1343-3p inhibitor was evidenced by the downregulation of Bax and the upregulation of Bcl-2; however, this phenomenon was reversed by ASMTL-AS1 silencing in HCC cells (Figure 4(b)). Additionally, the increased number of migrating HCC cells caused by treatment with the miR-1343-3p inhibitor was abrogated by ASMTL-AS1 silencing (Figure 4(c)). Collectively, ASMTL-AS1 acts as a sponge for miR-1343-3p to promote HCC cell proliferation and migration.

**Figure 4.** MiR-1343-3p inhibitor abrogates the deceleration of HCC cell proliferation and migration caused by ASMTL-AS1 silence. HCCLM3 and Huh cells transfected with si-NC, si-ASMTL-AS1, miR-1343-3p inhibitor, inhibitor NC, si-ASMTL-AS1+ miR-1343-3p inhibitor. a. Proliferation test by CCK8 assay. b. Western blot detection of Bcl-2 and Bax. d. Migration was assessed using transwell migration assays. * P < 0.05,** P < 0.001,vs.Si-NC; #P < 0.05, ## P < 0.001, vs.inhibitor-NC; ΔP<0.05, ΔΔP<0.001, vs. si-lnc+inhibitor.

### LAMC1 is the target of miR-1343-3p

As indicated above, LAMC1 is a downstream effector of ASMTL-AS1/miR-1343-3p ceRNA activity. The direct binding between LAMC1 and miR-1343-3p was predicted using starBase analysis (Figure 5(a)). To validate the interaction between LAMC1 and miR-1343-3p, LAMC1 3ʹ-UTR WT or LAMC1 3ʹ-UTR MUT were simultaneously transfected to HCCLM3 and Huh7 cells with miR-1343-3p mimic or mimic NC. Our results demonstrated that the miR-1343-3p mimic weakened the luciferase activity of LAMC1 3ʹ-UTR WT but not of LAMC1 3ʹ-UTR MUT. These data indicate the interplay between LAMC1 and miR-1343-3p (Figure 5(b)). Next, we tested LAMC1 expression in HCC tissues and found that LAMC1 mRNA was highly expressed in HCC tissues (Figure 5(c)). Interestingly, LAMC1 expression was negatively associated with miR-1343-3p expression and positively correlated with ASMTL-AS1 expression (Figure 5(d)). LAMC1 expression was higher in HCCLM3 and Huh7 cells than in THLE2 cells (Figure 5(e)). To determine whether miR-1343-3p interferes with LAMC1 expression, we transfected the miR-1343-3p inhibitor, si-LAMC1, or NCs into HCC cells. Western blot analysis showed that the miR-1343-3p inhibitor rescued LAMC1 expression in HCC cells (Figure 5(f)). In other words, miR-1343-3p targets the 3ʹ-UTR of LAMC1 and eventually downregulates LAMC1 expression. In addition, the downregulation of LAMC1 was a consequence of ASMTL-AS1 silencing in HCC cells (Figure 5(g)), suggesting that the transfection of si-ASMTL-AS1 curbed LAMC1 expression.

**Figure 5.** LAMC1 is the target of miR-1343-3p. a. Schematic representation of two potential binding sites of miR-1343-3p on LAMC1 3ʹUTR. b. The relative luciferase activity of miR-1343-3p mimics or NC on the luciferase reporter plasmid with wild type LAMC1 3ʹUTR sequence (WT) or both mutant binding sites of LAMC1 3ʹUTR (Mutation) was detected in HCCLM3 and Huh7 cells. c. qRT-PCR examined the LAMC1 expression in HCC tissues and normal tissues. d. Pearson correlation analysis between miR-1343-3p expression or ASMTL-AS1 and LAMC1 expression in HCC tissues. e. qRT-PCR examined the LAMC1 expression in HCCLM3, Huh7, and THLE3 cells. f. Western blots examined the LAMC1 protein expression in HCCLM3 and Huh7 transfected with si-NC, si-LAMC1, miR-1343-3p inhibitor, inhibitor NC and si-LAMC1+ miR-1343-3p inhibitor. *P < 0.05, **P < 0.001, vs.Si-NC; # P < 0.05, ## P < 0.001, vs. inhibitor-NC; ΔP<0.05,ΔΔP<0.001,vs. si-LAMC1+ inhibitor. g. Western blots examined the LAMC1 protein expression in HCCLM3 and Huh7 transfected with si-NC, si- ASMTL-AS1, **P < 0.001, vs. Si-NC.

### LAMC1 silencing attenuates the accelerated oncogenic phenotypes of HCC cells caused by the miR-1343-3p inhibitor

Considering the interaction between miR-1343-3p and LAMC1, we examined whether miR-1343-3p exerts its role by downregulating LAMC1 expression. As expected, LAMC1 silencing conferred proliferation defects on HCC cells, and the proliferation advantage conferred by the miR-1343-3p inhibitor was reversed upon LAMC1 knockdown (Figure 6(a)). Meanwhile, Western blotting detected elevated Bax expression in addition to reduced Bcl-2 expression in LAMC1-silenced HCC cells, suggesting that LAMC1 knockdown triggers HCC cell apoptosis. However, the pro-apoptotic effect of LAMC1 knockdown was counteracted by the miR-1343-3p inhibitor (Figure 6(b)). Additionally, the quantification of HCC cell migration illustrated that the migratory rate of HCC cells after LAMC1 silencing was considerably reduced, and this inhibition exerted by LAMC1 silencing was almost nullified by the miR-1343-3p inhibitor. This shows that the migratory capacity of HCC cells co-transfected with miR-1343-3p inhibitor and si-LAMC1 was comparable to that of the NC-treated groups (Figure 6(c)). These findings highlight that miR-1343-3p targets 3ʹUTR LAMC1 and weakens the oncogenic role of LAMC1.

**Figure 6.** LAMC1 silence attenuates the accelerated proliferation and migration of HCC cells caused by miR-1343-3p inhibitor. HCCLM3 and Huh7 were transfected with si-NC, si-LAMC1, miR-1343-3p inhibitor, inhibitor NC and si-LAMC1+ miR-1343-3p inhibitor. After 48 h transfection, a. CCK8 to detect cell proliferation change. b. Western blot and Western blot analysis of Bax and Bcl-2 protein expression. c. Migration was assessed using transwell migration assays. *P < 0.05, **P < 0.001, vs.Si-NC; # P < 0.05, ## P < 0.001, vs. inhibitor-NC; ΔP<0.05,ΔΔP<0.001, vs. si-LAMC1+ inhibitor.

## Discussion

Accumulating evidence has indicated the involvement of lncRNAs in governing malignant behaviors [19]. In the present study, ASMTL-AS1 was observed to be highly expressed in HCC tissues and cells. Loss of function studies in HCC cells illustrated that ASMTL-AS1 silencing caused HCC cell proliferation and migration, in addition to triggering apoptosis. Mechanistic analysis indicated that ASMTL-AS1 sequestered miR-1343-3p and rescued the interference of miR-1343-3p with LAMC1, subsequently promoting HCC progression.

Recently, ASMTL-AS1 was reported to be abnormally expressed in breast cancer, bladder cancer, thyroid carcinoma, and HCC [10–12]. However, its role in cancer may be context-dependent. For example, in breast cancer, the poor expression of ASMTL-AS1 was tightly linked with advanced stage and poor prognosis, and ASMTL-AS1 overexpression might inactivate the oncogenic Wnt/β-catenin pathway and subsequently retard breast cancer progression *in vitro* and *in vivo* [11]. In papillary thyroid carcinoma, ASMTL-AS1 exerts tumor-suppressive functions by suppressing the proliferative and metabolic phenotypes of tumor cells [10]. However, Qing et al. applied a TCGA BLCA cohort in bladder cancer and identified ASMTL-AS1 as an extracellular matrix-related lncRNA that might be a dismal prognostic signature. Interestingly, ASMTL-AS1 is highly expressed in HCC and exerts its oncogenic role by activating YAP signaling [12]. To further confirm the role of ASMTL-AS1 in HCC, we first detected its expression in HCC tissues and cells. Consistent with previous investigations, ASMTL-AS1 was amplified in HCC. Subsequent functional assays also demonstrated that ASMTL-AS1 silencing inhibited HCC cell proliferation and migration. The *in vitro* findings were corroborated *in vivo*. Therefore, our findings support the notion that ASMTL-AS1 is a tumor suppressor in HCC.

Previously, ASMTL-AS1 was reported as a ceRNA for miR-342-3p that activates the YAP signaling pathway in HCC [12]. Notably, ceRNA crosstalk frequently occurs because each lncRNA can target different miRNAs and may establish a complex ceRNA regulatory network. In the present study, starBase analysis demonstrated that several miRNAs, including miR-342-3p, shared a putative binding site with ASMTL-AS1; hence, we focused on miR-342-3p expression. MiR-342-3p has a tumor-suppressive role in various cancers, such as ovarian carcinoma [20] and hepatocellular carcinoma [21]. In HCC, miR-342-3p inhibits glycolysis and remodels tumor cell metabolism, a typical cancer hallmark [12]. It also negatively modulates the NF-κB pathway and inhibits HCC progression [22]. Consistently, our data showed that miR-342-3p was downregulated in HCC tissues and cells and that anti-miR-342-3p treatment resulted in an increase in HCC cell proliferation and migration. However, its upstream regulatory network has not yet been addressed. To find evidence supporting the interaction of miR-342-3p and ASMTL-AS1, luciferase reporter assays and RNA RIP assays were performed to confirm the direct targets of miR-342-3p and ASMTL-AS1. Furthermore, treatment with a miR-342-3p inhibitor rescued the proliferative and migratory defects of HCC cells after ASMTL-AS1 silencing. The negative correlation between miR-342-3p and ASMTL-AS1 in HCC tissues also supports this ceRNA activity. Therefore, ASMTL-AS1 might sponge miR-342-3p to repress its tumor-suppressor role in HCC and promote cancer progression.

The *LAMC1* gene is located on chromosome 1q25.3 and consists of 28 exons. It encodes a family of extracellular matrix glycoproteins characterized by a cruciform structure consisting of three short arms. It has been implicated in various oncogenic biological processes and functions as a tumor promoter in different cancers [23–25]. LAMC1 was enriched in HCC tissues and was defined as an unfavorable prognostic signature; silencing of *LAMC1* can strengthen the malignant behavior of HCC cells *in vitro* [26]. In line with previous investigations, we also found that LAMC1 knockout increased the proliferation and migration of HCC cells. Interestingly, we found that *LAMC1* is also a target of miR-1343-3p. Treatment with a miR-1343-3p inhibitor can counteract the effect of *LAMC1* silencing on HCC cell proliferation and migration. In addition, ASMTL-AS1 silencing resulted in the reduced expression of LAMC1 in HCC cells, suggesting that ASMTL-AS1 silencing might aggravate the inhibition of miR-1343-3p on LAMC1 expression. The ceRNA regulatory network hypothesis was further supported by the finding that LAMC1 expression was negatively correlated with miR-1343-3p expression and positively associated with ASMTL-AS1 expression in HCC tissues. Therefore, ASMTL-AS1 might rescue LAMC1 expression from miR-1343-3p-mediated inhibition, eventually favoring HCC progression.

However, this study has some limitations. First, *in vivo* assays were performed to validate our findings. Second, ASMTL-AS1 might have a more complex ceRNA network to regulate HCC progression because it has different targets. Moreover, this study only used GEPIA to identify key mRNAs in HCC. The key mRNAs or miRNAs might be screened out by other databases, such as the GEO DataSets and TCGA, which need further exploration. In addition, more clinical cases should be included to validate the expression of the indicated genes.

## Conclusion

In conclusion, our study provides evidence that ASMTL-AS1 is enriched in HCC tissues and cells. Mechanistically, ASMTL-AS1 acts as a ceRNA for miR-1343-3p and might release LAMC1 from miR-1343-3p, promoting HCC progression. Therefore, targeting the ASMTL-AS1/miR-1343-3p/LAMC1 axis may provide a novel therapeutic approach for the treatment of HCC.

## Data Availability

The datasets used and/or analyzed during the current study are available from the corresponding author on reasonable request.

## Highlights

- ASMTL-AS1 downregulation inhibits HCC progression *in vitro* and *in vivo*.
- ASMTL-AS1 could sponge miR-1343-3p to enhance LAMC1 expression.

ASMTL-AS1 targets the miR-1343-3p/LAMC1 axis to inhibit HCC malignant behavior.
